The article "Inhibitory effects of aromatase inhibitor on estrogen receptor-alpha positive ovarian cancer in mice" was published in 2014. Journal: J Ovarian Res.

# Inhibitory effects of aromatase inhibitor on estrogen receptor-alpha positive ovarian cancer in mice

**DOI:** 10.1186/1757-2215-7-4

**Published:** 2014-01-10

**Authors:** Hachidai Hirakawa, Yoshihito Yokoyama, Hidemi Yoshida, Hideki Mizunuma

**Affiliations:** 1 Department of Obstetrics and Gynecology, Hirosaki University Graduate School of Medicine, 5 Zaifu-cho, Hirosaki, Aomori 036-8261, Japan; 2 Department of Vascular Biology, Institute of Brain Science, Hirosaki University Graduate School of Medicine, 5 Zaifu-cho, Hirosaki, Aomori 036-8562, Japan

**Keywords:** Recurrent ovarian cancer, Letrozole, Estrogen receptor alpha, Aromatase inhibitor, Anti-angiogenesis

## Abstract

**Background:**

Estrogen causes proliferation of ovarian cancer cells. Although hormone therapy with an anti-estrogen agent is an optional therapy for recurrent epithelial ovarian cancers, both basic and clinical researches are insufficient. We here examine the efficacy of an aromatase inhibitor (AI) for peritonitis carcinomatosa, the late stage of ovarian cancer.

**Methods:**

Estrogen receptor (ER)α was assayed in four ovarian cancer cell lines by the RT-PCR method. Using ovariectomized nude mice, peritonitis carcinomatosa consisting of OVCAR-3 cells with the strongest ERα expression or DISS cells with weaker ERα expression was prepared. The survival period was compared between the letrozole group (5 mg/kg/day orally; n = 10) and the control group (n = 10). In addition, the degree of angiogenesis and occurrence of apoptosis were compared using tumor tissue from the abdominal cavity. The expression of aromatase and the protein involving in ERα signaling were examined in tumors immunohistochemically.

**Results:**

Survival period in OVCAR-3 tumors was significantly prolonged in the letrozole group, compared with the control group (*P* < 0.05), whereas that in DISS tumors was not different between the both groups. The microvessel density in tumors and expression of VEGF decreased significantly in the letrozole group compared to the control group. The incidence of apoptosis did not differ significantly between these groups. No adverse event was observed accompanying the administration of letrozole. The expressions of aromatase, ERα and FOXP1 that is associated with ERα signaling were reduced in tumors by letrozole administration.

**Conclusions:**

Letrozole was effective for ovarian cancers with abundant expression of ERα. Inhibition of angiogenesis and of ascites production appeared to contribute to prolongation of the survival period.

## Background

Ovarian cancer is still the most lethal of all gynecologic cancers. The American Cancer Society estimated that about 22,240 new cases of ovarian cancer will be diagnosed and 14,030 women will die of ovarian cancer in the United States in 2013 [1]. There are various methods for treating of recurrent ovarian cancer and chemotherapeutic regimen is chosen based on platinum susceptibility but there is no established second-line therapy.

In the National Comprehensive Cancer Network (NCCN) guidelines (version 3, 2012), hormone therapy is classified under “other drugs that are potentially effective” as “approved treatment for recurrent forms” of epithelial ovarian cancer. However, the number of clinical and basic studies of hormone therapy conducted for this disease is insufficient.

There is evidence that estrogen promotes proliferation of ovarian cancer in cell culture and a xenograft model [2-6]. Furthermore, it has been shown that the growth of ovarian cancer cells is inhibited *in vivo* and *in vitro* by the anti-estrogen therapy directed at estrogen receptor (ER) positive OVCAR-3 cells [3,5,6].

There are two types of ERα and ERβ. ERα is expressed in up to 60% of ovarian cancers [7]. ERα activates expression of genes that are involved in cell survival and proliferation, whereas the function of ERβ has been found to be anti-proliferative [8]. Because the growth response in ovarian cancer cell lines is mediated by ERα but not by ERβ [5,9], treatment with an ERα specific agonist (PTT,4′,4′,4″- (4-(4-Propyl-[1H]-pyrazole-1,2,5-tryl)trisphenol) promotes cell proliferation [5].

Aromatase converts adrenal androstenedione to estrogen and is expressed in fat, liver, muscle and cancers such as the breast and the ovary [10]. Intra-tumoral estrogens derived from *in situ* aromatization act as an autocrine growth factor that promotes cancer cell proliferation independent of circulating estrogen [11]. Aromatase inhibitors (AIs) inhibit estrogen production in postmenopausal women by more than 90%. Expression of aromatase mRNA and the aromatase protein itself have been found in 33-81% of ovarian cancers [12,13].

The therapeutic effect of AIs has been shown to be superior to that of tamoxifen as adjuvant therapy for breast cancer [14]. In addition, *in vitro* studies showed an anti-tumor effect of AI on ovarian cancer cells, which was associated with aromatase activity and ER expression [15]. Letrozole is an oral non-steroidal AI and used for the treatment of local or metastatic breast cancer that is ER positive.

The present study was conducted to evaluate the efficacy of letrozole in the late stages of ERα positive ovarian cancer and elucidate the mechanism.

## Methods

### Cell cines and cell culture

OVCAR-3 derived from human ovarian papillary adenocarcinoma and TOV-112D derived from human ovarian endometrioid adenocarcinoma were obtained from the American Type Culture Collection (Rockville, MD). MCAS derived from human ovarian mucinous adenocarcinoma was obtained from Japanese Collection of Research Bioresources Cell Bank (Osaka, Japan). DISS derived from human ovarian serous adenocarcinoma was kindly provided by Dr. Saga (Jichi Medical School, Tochigi, Japan) [16]. All of these cell lines were grown in RPMI 1640 medium supplemented with 10% fetal bovine serum, 100 U/ml penicillin and 100 μg/ml streptomycin at 37°C in a water-saturated atmosphere with 5% CO_2_/95% air. All cell lines used in this study are authenticated as being ovarian in origin with a written guarantee.

### Animal experimentation

Animal experiments were conducted in accordance with the Guidelines for Animal Experimentation, Hirosaki University. Eight-week-old female BALB/c nu/nu mice were used in this study. At the Institute for Animal Experimentation of Hirosaki University, all mice were group-housed in plastic cages with stainless-steel grid tops, under a 12-hour light dark cycle and consumed water and food ad libitum.

### Hormone administration and ovariectomy

Letrozole was purchased from Novartis Oncology (Tokyo, Japan). Letrozole was suspended in distilled water (0.88 mmol/l). The experimental mice were divided into two groups containing ten mice each. The letrozole group was given letrozole 5 mg/kg/day by oral gavage every day until the end of the study, and the control group was given vehicle. Bilateral ovariectomy was performed under pentobarbital anesthesia in all experimental mice on the seventh day after commencement of letrozole administration.

### Real-time quantitative PCR

Total RNA was extracted from the cells using an Illustra RNAspin Mini RNA Isolation Kit (GE Healthcare, Piscataway, NJ). Total RNA (4 μg) served as a template for single-strand cDNA synthesis in a reaction using an iScript Advanced cDNA Kit (Bio-Rad, Hercules, CA) under the conditions [17] with slight modifications. A CFX96 real-time PCR detection system (Bio-Rad) was used for the quantitative analyses of ERα and glyceraldehyde-3-phosphate dehydrogenase (GAPDH). The sequences of the primers were as follows:

ERα-F (5′-TGGGCTTACTGACCAACCTG-3′),

ERα-R (5′-CCTGATCATGGAGGGTCAAA-3′),

GAPDH-F (5′-ACCACCAACTGCTTAGCACC-3′), and

GAPDH-R (5′-CCATCCACAGTCTTCTGGGT-3′).

The amplification reactions were performed with SsoFast EvaGreen Supermix (Bio-Rad) according to the manufacturer’s specifications. The primers were used at 300 nM. The amplification conditions were as follows: 30 sec at 95°C, followed by 95°C for 5 sec and 60°C for 30 sec for 40 consecutive cycles. After amplification, a melting curve 65°C to 95°C at 0.5°C increments and 5 sec per step was generated with continuous monitoring of fluorescence. The melting curves and quantitative analysis of the data were performed using CFX manager Version 2.1 software (BioRad) [17].

### Evaluation of adverse effects following administration of letrozole

The nude mice, ovariectomized at the age of nine weeks were given letrozole (n = 10) or its vehicle (n = 10) for five weeks. All mice were weighed every day and the consumption of food was measured daily. Acts of self-harm or aggression were also observed.

### Mouse model of peritoneal carcinomatosis

OVCAR-3 cells (5.0 × 10^6^ cells) or DISS cells (5.0 × 10^6^ cells) were inoculated into the peritoneal cavity of ovariectomized nude mice in 500 μl of RPMI 1640 medium at the age of nine weeks. The survival times for the letrozole and control groups were evaluated. The survival was compared until 5 weeks after cell inoculation and surviving mice were euthanized using high-dose pentobarbital in order to remove the peritoneal tumors for histologic and biochemical evaluation.

### Immunohistochemical analysis and microvessel density

Six-micrometer sections of formalin-fixed and paraffin-embedded tissue specimens were stained by an established method described previously [18]. Sections were incubated with antibodies specific for Factor VIII (DAKO, Tokyo, Japan), vascular endothelial growth factor (VEGF) (R & D Systems, Minneapolis, MN), cleaved caspase-3 (Santa Cruz Biotechnology, Santa Cruz, CA), human P450 aromatase (ARK Resource, Kumamoto, Japan), ERα (Santa Cruz Biotechnology) and FOXP1 (Abcam, Tokyo, Japan) at 4°C overnight. Slides were incubated with biotinylated species-specific appropriate secondary antibodies for 30 minutes and exposed to avidin-biotin-peroxidase complex (VECTA Laboratories, Burlingame, CA). Sections were treated with 0.02% DAB as a chromogen and counterstained with hematoxylin. Microvessel density (MVD) was determined as follows. The highly vascularized areas of the tumor stained with an anti-Factor VIII antibody were identified and Factor VIII-positive microvessels were counted within a high-power field (number per 0.75 mm^2^). Single endothelial cells or clusters of endothelial cells, with or without lumen, were considered individual vessels. MVD was expressed as the vessel number/high-power field in sections. Three fields were counted per animal and the average was taken as the MVD of each tumor.

### Weatern blot analysis

Cell lysates (50 μg protein) were prepared from tumor tissues, electrophoresed through a 12.5% SDS-polyacrylamide gel, and blotted as described previously [18]. The protein concentration was determined using Bradford’s method. The blots were probed with the following diluted antibodies for 2 hr: cleaved caspase-3 (active, 17KDa) at 1:1000 and β-actin (Sigma-Aldrich, St Louis, MO) at 1:2000. The membranes were then incubated for 1 hr with the appropriate biotinylated secondary antibodies, transferred to avidin-biotin-peroxidase complex reagent, and incubated in this solution for 30 min. Diaminobenzidine (Sigma-Aldrich) was used as a substrate.

### Statistical analysis

Survival rates were calculated by the Kaplan-Meier method, and the statistical significance of differences in the cumulative survival curves between the groups was evaluated using the log-rank test. Other statistical analysis was carried out with the Student *t*-test. A result was deemed significant at a *P* value < 0.05.

## Results

### Comparison of mRNA expression of ERα in the ovarian cancer cell lines

We determined mRNA abundance of ERα in four ovarian cancer cell lines using real-time quantitative PCR. We found that the level of ERα mRNAin OVCAR-3 cells was significantly higher than that in other three cell lines (*P* < 0.05, Figure 1). Thus, OVCAR-3 was defined as ERα positive, whereas DISS, MCAS and TOV-112D were defined as ERα negative.

**Figure 1:** **Determination of estrogen receptor-alpha (ERα) mRNA level in four ovarian cancer cell lines.** The level of ERα mRNA was significantly higher in OVCAR-3 cells in comparison to the other three lines. ERα mRNA expression was normalized to GAPDH mRNA expression (DISS as control = 1). Means ± SD of three experiments are shown. * *P* < 0.05 versus OVCAR-3.

### Evaluation of adverse effect caused by giving letrozole after ovariectomy

Changes in the body weights of ovariectomized mice were evaluated. Body weights were 27.9 ± 1.4 in mice given letrozole for 5 weeks and 28.1 ± 2.4 in mice given vehicle, with no significant difference. All of the mice were healthy and did not exhibit self-harm or act aggressively.

### Comparison of survival period in peritonitis carcinomatosa derived from OVAR-3 cells or DISS cells

Survival times were compared between the letrozole and the control groups in the peritonitis cacinomatosa (Figure 2A). Survival periods in ERα positive OVCAR-3 tumors were significantly prolonged in the letrozole group, compared with the control group (*P* < 0.05, Figure 2B), whereas those in ERα negative DISS tumors were not different between the both groups (Figure 2C).

**Figure 2:** **Comparison of the survival period in the letrozole group and the control group. (A)** Appearances, intraperitoneal finding and bloody ascites of peritoneal carcinomatosa mice model derived from OVCAR-3 cells. Asterisks show disseminated foci of the cancer. **(B)** The survival period in the letrozole group was extended significantly beyond that in the control group in ERα positive OVCAR-3 tumors (*P* < 0.05). **(C)** There was no signicant difference in survival period between the groups in ERα negative DISS tumors.

### Altered expression of aromatase, ERα and FOXP1 in tumors by letrozole

We compared aromatase expression in tumors in order to examine whether letrozole administration affects *in situ* aromatization. Expressions of ERα and FOXP1 involving in ERα signaling [19] were also examined. Immunohistochemical analysis showed that expression of aromatase, ERα and FOXP1 in tumors was reduced by letrozole administration (Figure 3).

**Figure 3:** **Comparison of expression of aromatase, ERα and FOXP1 in tumors between the control and letrozole groups.** Immunohistochemical staining shows descreased expression of aromatase, ERα and FOXP1 by letrozole administration, compared to the control.

### Reduction of microvessel density and VEGF level in tumors by letrozole

We examined the number of microvessels identified in tumor tissues using an immunostaining method for Factor VIII. MVD (number/mm^2^) was 8.9 ± 1.4 for the control group, and 5.8 ± 1.8 for the letrozole group, showing a significant decrease in the letrozole group as compared with the control group (*P* < 0.05, Figure 4A). Immunostaining showed a notable decrease in the expression of VEGF in tumors in the letrozole group, as compared with the control group (Figure 4B).

**Figure 4:** **Comparison of microvessel density (MVD) and VEGF expression in the letrozole group and the control group. (A)** The MVD in the letrozole group was significantly lower than that in the control group. * *P* < 0.05. **(B)** VEGF expression in the letrozole group was remarkably lower than that in the control group.

### Comparison of apoptotic cells identified with caspase-3 antibody and expression of caspase-3

The number of apoptotic cells per mm^2^ was 320 ± 32 in the control group, and 272 ± 32 in the letrozole group, an insignificant difference between the groups (Figure 5A). Western blot also showed no significant difference of expressions of caspase-3 between the groups (Figure 5B).

**Figure 5:** **Apoptotic cells identified with caspase-3 antibody and expression of caspase-3. (A)** Immunohistochemical staining. Brown-colored cells are an apoptotic cell identified with caspase-3 antibody. **(B)** Western blot. There is no significant difference in expressions of caspase-3 between the groups.

## Discussion

In this study, we prepared a model of peritonitis carcinomatosa, using ovariectomized nude mice and examined the effect of an AI on this condition, which occurs most frequently as a mode of postoperative recurrence of ovarian cancer. We found that the survival was extended significantly by the administration of letrozole in peritonitis carcinomatosa produced by inoculation of OVCAR-3 that exhibited strongest ERα expression. As regards the mechanism of action, decreases in MVD and VEGF expression suggested that inhibition of both angiogenesis and production of ascites contributed to prolongation of survival.

It has been reported that VEGF plays an important role in angiogenesis and ascites production and the expression of VEGF is regulated by estrogen [20]. Presence of an estrogen-responsive element was established for the VEGF gene [21], and the contribution of estrogen to a direct increase in expression of the VEGF gene and angiogenesis has been demonstrated [22]. These results therefore indicate that estrogen accelerates tumor progression by means of VEGF. Conversely, AIs are shown to decrease the estrogen level in breast cancer tissues [23] and reduce VEGF in breast cancer cells [24]. The present study shows for the first time that the administration of an AI decreased VEGF and MVD in OVCAR-3 that is derived from ovarian cancer. The present results provide evidence for inhibition of angiogenesis by the AI and indicate that inhibition of angiogenesis is the mechanism by which AIs suppress tumor proliferation. In breast cancers, estrogen and ER are involved in tumor proliferation and tumor proliferation is inhibited by the anti-estrogen activity [25]. Although it has not been shown in ovarian cancers that estrogen and ER are involved in tumor proliferation in a similar manner to breast cancers, an effect of AIs on ER-positive ovarian cancer can be expected based on the results of this study, which demonstrated inhibition of tumor proliferation in ERα-positive ovarian cancers by the AI. In this study, expression of aromatase, ERα and FOXP1 in OVCAR-3 tumors was reduced by letrozole administration. Aromatization of androstendione may be inhibited in OVCAR-3 tumors by letrozole. FOXP1 is situated at a downstream of ERα signaling [19]. These results suggest that suppression of aromatization and ERα signaling in ERα-positive ovarian cancer by the AI may contribute to inhibition of tumor proliferation.

*In vitro* experiments using breast cancer cells have shown an induction of apoptosis by AIs [26], indicating that this is the mechanism of inhibition of breast cancer proliferation. AIs have also been reported to increase *in vivo* apoptosis significantly in combination with an mTOR inhibitor, thereby exhibiting an anti-tumor effect [27]. Amarai et al. have emphasized the importance of AIs as inducers of apoptosis, by effects on both mitochondria and caspase-8 [28]. On the other hand, Bailey et al. have reported that the combination of an AI and an apoptosis inducer is an effective treatment strategy for ER-positive breast cancers, as ERs inhibit p53-induced apoptosis but AIs block the signaling of ERs [29]. Thus, AIs were shown to produce an environment favorable to apoptosis by inhibiting the activity of ERs, although they did not inhibit apoptosis directly [29]. The results of our study, which did not show a significant increase in apoptosis in ovarian tumors following the administration of an AI, agree with the results of Bailey et al.

AIs have been shown to be more effective than tamoxifen if they are used as postoperative adjuvant therapy in breast cancers [30]. No definite conclusion, however, has yet been reached with regard to the effect of AIs in recurrent ovarian cancers. The effects of AIs on *in vitro* ovarian cancer cells were related to aromatase activity and estrogen receptor expression [6]. Of four clinical studies that have verified the efficacy of letrozole in recurrent ovarian cancers [31-34], three clinical studies conducted in patients with ERα-positive recurrent ovarian cancers showed that the response rate to letrozole was 11.8% in the 102 patients [31-33]. However, the details of progression-free survival or overall survival are unknown. Adverse reactions to letrozole were slight compared to those of anticancer agents and the response rate of 11.8% is similar to that obtained with salvage chemotherapy. As shown in Figure 3, letrozole has an inhibitory effect on angiogenesis, therefore it is expected that patients with ERα-positive recurrent ovarian cancers are candidates of letrozole administration alone or in combination with bevacizumab, a drug that targets molecules involved in angiogenesis.

Estrogen accelerates angiogenesis and is involved in the progression of tumors [35]. ER signaling inhibits apoptosis [29]. Letrozole, an AI, has been shown to exhibit an antitumor effect by inhibiting angiogenesis in ERα-positive ovarian cancers and by inhibiting the actions of ERα. Although the effect of letrozole on survival was statistical significant in mice, it is an important issue whether the clinical significance of the findings will be achieved. Thus, further investigation of whether Letrozole sensitizes OVCAR-3 tumour to platinum compound is warranted. AIs will likely play a central role in the establishment of a new treatment strategy in ERα-positive ovarian cancers in the future. Clinical trials of letrozole alone or in combination with other molecular targeted drugs will be required to further evaluate the drug’s efficacy in the treatment of ERα-positive ovarian cancers.

## Conclusions

Letrozole was effective for peritonitis carcinomatosa as a late stage of ovarian cancer with abundant expression of ERα. Inhibition of angiogenesis and of ascites production appeared to contribute to prolongation of the survival period.

## Abbreviations

ER: Estrogen receptor; AI: Aromatase inhibitor; VEGF: Vascular endothelial growth factor; MVD: Microvessel density.

## Competing interests

The authors declare that they have no competing interest.

## Authors’ contributions

HH and YY conceived and designed the study, performed the experiments and wrote the paper. HM contributed to the writing and to the critical reading of the paper. HY performed RT-PCR experiment as a coach and contributed to the critical reading of the paper. All authors read and approved the final manuscript.

## References

[B1] SiegelRNaishadhamDJemalACancer statistics, 2013CA Cancer J Clin2013631113010.3322/caac.2116623335087

[B2] LangdonSPHirstGLMillerEPHawkinsRATesdaleALSmythJFMillerWRThe regulation of growth and protein expression by estrogen *in vitro*: a study of 8 human ovarian carcinoma cell linesJ Steroid Biochem Mol Biol1994503–4131135804914110.1016/0960-0760(94)90019-1

[B3] LangdonSPCrewAJRitchieAAMuirMWakelingASmythJFMillerWRGrowth inhibition of oestrogen receptor-positive human ovarian carcinoma by anti-oestrogens *in vitro* and in a xenograft modelEur J Cancer199430A5682686808068810.1016/0959-8049(94)90545-2

[B4] Armaiz-PenaGNMangalaLSSpannuthWALinYGJenningsNBNickAMLangleyRRSchmandtRLutgendorfSKColeSWSoodAKEstrous cycle modulates ovarian carcinoma growthClin Cancer Res20091592971297810.1158/1078-0432.CCR-08-252519383821PMC2743312

[B5] SimpkinsFHevia-PaezPSunJUllmerWGilbertCAda SilvaTPedramALevinERReisIMRabinovichBAzzamDXuXXInceTAYangJYVerhaakRGLuYMillsGBSlingerlandJMSrc inhibition with saracatinib reverses fulvestrant resistance in ER-positive ovarian cancer models *in vitro* and *in vivo*Clin Cancer Res201218215911592310.1158/1078-0432.CCR-12-125722896656PMC3698880

[B6] SimpkinsFGarcia-SotoASlingerlandJNew insights on the role of hormonal therapy in ovarian cancerSteroids201378653053710.1016/j.steroids.2013.01.00823402742PMC4551472

[B7] PujolPReyJMNirdePRogerPGastaldiMLaffargueFRochefortHMaudelondeTDifferential expression of estrogen receptor-alpha and -beta messenger RNAs as a potential marker of ovarian carcinogenesisCancer Res19985823536753739850067

[B8] BardinAHoffmannPBoulleNKatsarosDVignonFPujolPLazennecGInvolvement of estrogen receptor beta in ovarian carcinogenesisCancer Res200464165861586910.1158/0008-5472.CAN-04-055215313930

[B9] O’DonnellAJMacleodKGBurnsDJSmythJFLangdonSPEstrogen receptor-alpha mediates gene expression changes and growth response in ovarian cancer cells exposed to estrogenEndocr Relat Cancer200512485186610.1677/erc.1.0103916322326

[B10] CunatSRabenoelinaFDaurèsJPKatsarosDSasanoHMillerWRMaudelondeTPujolPAromatase expression in ovarian epithelial cancersJ Steroid Biochem Mol Biol2005931152410.1016/j.jsbmb.2004.10.02115748828

[B11] LabrieFBelangerASimardJVanLLabrieCDHEA and peripheral androgen and estrogen formation: intracinologyAnn N Y Acad Sci1995774162810.1111/j.1749-6632.1995.tb17369.x8597456

[B12] SlotmanBJKuhnelRRaoBRDijkhuizenGHDeGJStolkJGImportance of steroid receptors and aromatase activity in the prognosis of ovarian cancer: high tumor progesterone receptor levels correlate with longer survivalGynecol Oncol1989331768110.1016/0090-8258(89)90607-02703171

[B13] KitawakiJNoguchiTYamamotoTYokotaKMaedaKUrabeMHonjoHImmunohistochemical localisation of aromatase and its correlation with progesterone receptors in ovarian epithelial tumoursAnticancer Res199616191978615676

[B14] WongZWEllisMJFirst-line endocrine treatment of breast cancer: aromatase inhibitor or antioestrogen?Br J Cancer2004901202510.1038/sj.bjc.660150814710200PMC2395329

[B15] SasanoHSatoSItoKYajimaANakamuraJYoshihamaMArigaKAndersonTJMillerWREffects of aromatase inhibitors on the pathobiology of the human breast, endometrial and ovarian carcinomaEndocr Relat Cancer19996219720410.1677/erc.0.006019710731109

[B16] YokoyamaYXinBShigetoTUmemotoMKasai-SakamotoAFutagamiMTsuchidaSAl-MullaFMizunumaHClofibric acid, a peroxisome proliferator–activated receptor α ligand, inhibits growth of human ovarian cancerMol Cancer Ther2007641379138610.1158/1535-7163.MCT-06-072217431116

[B17] MengPYoshidaHMatsumiyaTImaizumiTTanjiKXingFHayakariRDempoyaJTatsutaTAizawa-YashiroTMimuraJKosakaKItohKSatohKCarnosic acid suppresses the production of amyloid-β 1–42 by inducing the metalloprotease gene TACE/ADAM17 in SH-SY5Y human neuroblastoma cellsNeurosci Res20137529410210.1016/j.neures.2012.11.00723257508

[B18] SakamotoAYokoyamaYUmemotoMFutagamiMSakamotoTBingXMizunumaHClinical implication of expression of cyclooxygenase-2 and peroxisome proliferator activated-receptor gamma in epithelial ovarian tumoursBr J Cancer20049146336381526633310.1038/sj.bjc.6602009PMC2364772

[B19] RayooMYanMTakanoEABatesGJBrownPJBanhamAHFoxSBExpression of the forkhead box transcription factor FOXP1 is associated with oestrogen receptor alpha, oestrogen receptor beta and improved survival in familial breast cancersJ Clin Pathol2009621089690210.1136/jcp.2009.06516919622517

[B20] DabrosinCMargettsPJGauldieJEstradiol increases extracellular levels of vascular endothelial growth factor *in vivo* in murine mammary cancerInt J Cancer2003107453554010.1002/ijc.1139814520689

[B21] HyderSMNawazZChiappettaCStancelGMIdentification of functional estrogen response elements in the gene coding for the potent angiogenic factor vascular endothelial growth factorCancer Res200060123183319010866309

[B22] NakamuraJSavinovALuQBrodieAEstrogen regulates vascular endothelial growth/permeability factor expression in 7,12-dimethylbenz(a)anthracene-induced rat mammary tumorsEndocrinology19961371255895596894038810.1210/endo.137.12.8940388

[B23] BrodieAMSchwarzelWCShaikhAABrodieHJThe effect of an aromatase inhibitor, 4-hydroxy-4-androstene-3,17-dione, on estrogen-dependent processes in reproduction and breast cancerEndocrinology197710061684169510.1210/endo-100-6-1684404132

[B24] FersisNSmyczek-GargyaBArmeanuSGagulicEPanticLRelakisKFriedrichMWallwienerDChanges in vascular endothelial growth factor (VEGF) after chemoendocrine therapy in breast cancerEur J Gynaecol Oncol2004251455015053061

[B25] CoezyEBorgnaJLRochefortHTamoxifen and metabolites in MCF7 cells: correlation between binding to estrogen receptor and inhibition of cell growthCancer Res19824213173237053859

[B26] LisztwanJPornonAChenBChenSEvansDBThe aromatase inhibitor letrozole and inhibitors of insulin-like growth factor I receptor synergistically induce apoptosis in *in vitro* models of estrogen-dependent breast cancerBreast Cancer Res2008104R5610.1186/bcr211310.1186/bcr211318611244PMC2575527

[B27] LiuYZhangXLiuJHouGZhangSZhangJEverolimus in combination with letrozole inhibit human breast cancer MCF-7/Aro stem cells via PI3K/mTOR pathway: an experimental studyTumour Biolin press10.1007/s13277-013-1170-824014089

[B28] AmaralCVarelaCBorgesMTavares da SilvaERoleiraFMCorreia-da-SilvaGTeixeiraNSteroidal aromatase inhibitors inhibit growth of hormone-dependent breast cancer cells by inducing cell cycle arrest and apoptosisApoptosis201318111426143610.1007/s10495-013-0879-623842740

[B29] BaileySTShinHWesterlingTLiuXSBrownMEstrogen receptor prevents p53-dependent apoptosis in breast cancerProc Natl Acad Sci USA201210944180601806510.1073/pnas.101885810923077249PMC3497783

[B30] CuzickJSestakIBaumMBuzdarAHowellADowsettMForbesJFEffect of anastrozole and tamoxifen as adjuvant treatment for early-stage breast cancer: 10-year analysis of the ATAC trialLancet Oncol201011121135114110.1016/S1470-2045(10)70257-621087898

[B31] RamirezPTSchmelerKMMilamMRSlomovitzBMSmithJAKavanaghJJDeaversMLevenbackCColemanRLGershensonDMEfficacy of letrozole in the treatment of recurrent platinum- and taxane-resistant high-grade cancer of the ovary or peritoneumGynecol Oncol20081101565910.1016/j.ygyno.2008.03.01418457865

[B32] SmythJFGourleyCWalkerGMacKeanMJStevensonAWilliamsARNafussiAARyeTRyeRStewartMMcCurdyJManoMReedNMcMahonTVaseyPGabraHLangdonSPAntiestrogen therapy is active in selected ovarian cancer cases: the use of letrozole in estrogen receptor-positive patientsClin Cancer Res200713123617362210.1158/1078-0432.CCR-06-287817575226

[B33] PapadimitriouCAMarkakiSSiapkarasJVlachosGEfstathiouEGrimaniIHamilosGZorzouMDimopoulosMAHormonal therapy with letrozole for relapsed epithelial ovarian cancer. Long-term results of a phase II studyOncology200466211211710.1159/00007743615138362

[B34] BowmanAGabraHLangdonSPLessellsAStewartMYoungASmythJFCA125 response is associated with estrogen receptor expression in a phase II trial of letrozole in ovarian cancer: identification of an endocrine-sensitive subgroupClin Cancer Res2002872233223912114425

[B35] IyerVKlebbaIMcCreadyJArendtLMBetancur-BoisselMWuMFZhangXLewisMTKuperwasserCEstrogen promotes ER-negative tumor growth and angiogenesis through mobilization of bone marrow-derived monocytesCancer Res201272112705271310.1158/0008-5472.CAN-11-328722467173

